# Prediction of Lung Infection during Palliative Chemotherapy of Lung Cancer Based on Artificial Neural Network

**DOI:** 10.1155/2022/4312117

**Published:** 2022-01-10

**Authors:** Wei Guo, Guoyun Gao, Jun Dai, Qiming Sun

**Affiliations:** The Second People's Hospital of Wuhu, Wuhu, Anhui 230032, China

## Abstract

Lung infection seriously affects the effect of chemotherapy in patients with lung cancer and increases pain. The study is aimed at establishing the prediction model of infection in patients with lung cancer during chemotherapy by an artificial neural network (ANN). Based on the data of historical cases in our hospital, the variables were screened, and the prediction model was established. A logistic regression (LR) model was used to screen the data. The indexes with statistical significance were selected, and the LR model and back propagation neural network model were established. A total of 80 cases of advanced lung cancer patients with palliative chemotherapy were predicted, and the prediction performance of different model was evaluated by the receiver operating characteristic curve (ROC). It was found that age≧60 years, length of stay≧14 d, surgery history, combined chemotherapy, myelosuppression, diabetes, and hormone application were risk factors of infection in lung cancer patients during chemotherapy. The area under the ROC curve of the LR model for prediction lung infection was 0.729 ± 0.084, which was less than that of the ANN model (0.897 ± 0.045). The results concluded that the neural network model is better than the LR model in predicting lung infection of lung cancer patients during chemotherapy.

## 1. Introduction

At present, lung cancer is still the leading cause of death globally [1–3]. Patients with advanced lung cancer who have multiple systemic metastases are less likely to receive palliative chemotherapy, because there is no indication for targeted therapy after gene detection. Palliative chemotherapy is also the use of traditional chemotherapy drugs, but the purpose is not to treat cancer but to reduce the clinical symptoms of lung cancer patients. Palliative chemotherapy can prolong the life of patients and help them recover their daily life. Therefore, the drug dose of palliative chemotherapy will be lower than that of general chemotherapy [4–6].

In the study of complications and causes of death in cancer patients, infection-related causes of death are as high as 76% [7–9]. The causes of infection in patients with lung cancer during chemotherapy are complex, and there are various risk factors affecting the disease [10, 11]. There may be an interaction between some risk factors and multicollinearity, which seriously interferes with the prediction of infection [12]. With the development of artificial intelligence technology, the artificial intelligence (AI) algorithm represented by deep learning is gradually applied in various medical fields and has achieved better diagnostic energy efficiency [13–16]. Among them, the back propagation (BP) neural network model is widely used to establish a prediction model in medical diagnosis [17].

The study analyzed 80 patients with lung cancer who were hospitalized for chemotherapy, established a specific prediction model by using the risk factors that affect the lung infection during palliative chemotherapy, and made an evaluation and prediction of the possible infection in patients with lung cancer. According to the prediction results, the individual status and whether preventive intervention measures should be taken can improve patients' treatment effect and quality of life.

## 2. Materials and Methods

### 2.1. General Information

The data collection time was from January 2019 to December 2019. All hospitalized patients with advanced lung cancer confirmed by clinical, imaging, and pathology were collected in this period. The cases collected in the study were approved by the ethics committee of the Second People's Hospital of Wuhu, and all patients were informed to sign informed consent.

The following are the inclusion criteria: (1) the diagnosis of lung cancer was supported by imaging and pathological results (Figure 1), (2) palliative chemotherapy was used, (3) estimated survival time of patients was greater than three months, and (3) there is no communication barrier with medical staff.

The following are the exclusion criteria: (1) serious complications, (2) serious physical diseases, (3) mental diseases, and (4) application for withdrawal from the study.

Finally, 80 patients were selected as the research objects. They were 56 male and 24 female patients, aged 46-86 (68.32 ± 9.45) years. In the TNM stage, there are 13 cases of IIIA stage, 27 cases of IIIB stage, 32 cases of IIIC stage, and 8 cases of IV stage. There were 7 cases of small-cell lung cancer, 30 cases of adenocarcinoma, 37 cases of squamous cell carcinoma, and 6 cases of other cancers.

### 2.2. Source of Data

The chemotherapy patients diagnosed as lung cancer by tissue and cytology were randomly selected by a stratified sampling method from January 2016 to December 2018. The demographic characteristics are shown in Table 1. The hospital history data should be unified and detailed, and the information collected includes age, sex, smoking index (smoking index = number of smoking per day × number of years of smoking), TNM stage, pathological classification, basic diseases, chemotherapy cycle, chemotherapy plan, invasive operation, lung cancer surgery history, radiotherapy history, leukocyte and albumin, adverse reactions after chemotherapy, hormone that should be used, antibiotics, and hospitalization time.

### 2.3. Criteria of Pulmonary Infection

According to the diagnostic criteria of nosocomial pulmonary infection formulated by the American Thoracic Association, the selected patients had at least two or more of the following manifestations: (1) there were fever, cough, and expectoration after and chemotherapy; (2) fever, cough, and expectoration had occurred before chemotherapy, and the symptoms were aggravated after chemotherapy; (3) the pulmonary rales become more and more after chemotherapy; and (4) chest X-ray showed new or progressive infiltration.

### 2.4. Back Propagation Neural Network

ANN is divided into three layers: input layer, hidden layer, and output layer.  Figure 2 is the schematic diagram of the neural network. Perceptron is the basic unit of neural network. It is composed of weight W, offset B, and transfer function *g*(*x*).

The ANN algorithm is deduced and trained to obtain the training results.

We set the input layer as *a*_1_, the hidden layer as *b*_2_*b*_3_ ⋯ *b*_*n*−1_, and the output layer as *c*_*n*_. We let the value of each perceptron in the input layer be *a*_1*n*_(*n* = 1, 2, 3⋯), and the other layers are similar. We set the weight *w*_*ab*_^*k*^ as the weight between the *a*-th sensing unit of layer *K* and the *b*-th sensing unit of layer *K* + 1. The bias is *b*′. According to the perceptron principle, the bias can be used as a perceptron with a weight of 1 and a signal of *b*′ in the upper layer. Therefore, bias *b*′ is not considered in the following derivation.

The implemented neural network model has preoutput, back propagation, updating weights, and other parameters (Figure 3). The brief steps are as follows.

(Step 1) We set the input signal received by each unit of the input layer as *x*_1_*x*_2_*x*_3_ ⋯ *x*_*n*_ and assign a random value to *w*. According to the above process, a set of calculation results can be obtained at the output layer.
(Step 2) The error between the predicted value and the real value is calculated in reverse, and the relationship between the final error and the initial weight is calculated.
(Step 3) Use stochastic gradient descent to find the minimum value of error *E*.
(Step 4) By iterating and updating *W*, the training is completed and the prediction results are obtained.

For Step 1, the input value reaches the value ∑_*i*=1_*w*_*i*1_^1^*a*_1*i*_ of the first neural unit *b*_21_ of the hidden layer *b*_2_ through weight calculation, and the input signal value of *b*_21_ is *g*(∑_*i*=1_*w*_*i*1_^1^*a*_1*i*_) through the transfer function *g*(*x*).

(1) $$\begin{array}{c} \text{The output layer is }c_{nj}=g\left(\underset{i=1}{\sum }w_{ij}^{n-1}b_{\left(n-1\right)i}\right).. \end{array}$$

For Step 2, set the label as *d*_*mi*_(*i* = 1, 2, 3⋯) and substitute the hidden layer unit *c*_*nj*_*n*__ to obtain the relationship *E* between the error and the initial weight.

According to Step 4,

(2) $$\begin{array}{c} E=\frac{1}{2}\underset{j_{n}=1}{\sum }{\left(d_{{nj}_{n}-c_{{nj}_{n}}}\right)}^{2} \end{array}$$

set

(3) $$\begin{array}{c} k=\underset{j_{n-1}=1}{\sum }w_{j_{n-1}j_{n}}^{n-1}b_{{\left(n-1\right)}_{j_{\left(n-1\right)}}},\\ \frac{\delta E_{i}}{\delta w_{ij}^{n-1}}=\frac{\delta E_{i}\delta c_{ni}\delta k}{\delta c_{ni}\delta k\delta w_{ij}^{n-1}}, \end{array}$$

and then the function (4) can be obtained

(4) $$\begin{array}{c} \frac{\vartheta E_{i}}{\vartheta w_{ij}^{n-1}}=-c_{ni}b_{\left(n-1\right)i}\left(d_{ni}-c_{ni}\right)\left(1-c_{ni}\right), \end{array}$$

and the weight *w*_*ij*_^*n*−1^can be updated to obtain function

(5) $$\begin{array}{c} {\left(w_{ij}^{n-1}\right)}^{*}=w_{ij}^{n-1}-\eta^{*}\underset{i=1}{\sum }\frac{\vartheta E_{i}}{\vartheta w_{ij}^{n-1}}. \end{array}$$

### 2.5. Statistical Analysis

In this study, considering that the number of neurons is too large and the sample size is high, the infection of lung cancer during chemotherapy was taken as the dependent variable, and the univariate and multivariate logistic regression (LR) analysis was carried out to establish the prediction model. The LR and artificial neural network (ANN) prediction models were established, respectively, using the 400 patients from January 2016 to December 2018. The test set was the 80 patients from January 2019 to December 2019. The *Z* test was used to compare the area under the receiver operator characteristics (ROC) curve with 0.5 to test whether the model has predictive value; the *Z* test was used to compare the area under the ROC curve of the model to evaluate the predictive effect of the model. The construction of LR model and the drawing of ROC curve are completed by SPSS software; the ANN model is constructed by MATLAB software, and the simulation and verification of test samples are carried out.

## 3. Results

### 3.1. Logistic Regression Analysis

From the univariate and multivariate conditional logistic regression analysis, seven indexes have statistical significance: age≧60 years, length of stay≧14 d, lung cancer surgery history, combined chemotherapy, myelosuppression, diabetes, and hormone application (Table 2). In multivariate analysis, the cut point value of classification was 0.5, and the maximum number of iterations was 20. The LR model was established by using the partial maximum likelihood forward method. The expression was follows:

(6) $$\begin{array}{c} \text{Logit }\left(P\right)=-0.482+0.718\;\left(\text{age}\right)+1.3749\;\left(\text{length of stay}\right)+0.192\;\left(\text{surgery history}\right)+0.593\;\left(\text{combined chemotherapy}\right)-1.452\;\left(\text{myelosuppression}\right)+0.674\;\left(\text{diabetes}\right)+0.269\;\left(\text{hormone application}\right). \end{array}$$

### 3.2. ANN Analysis

According to the influence degree of input influencing factors on the network, the following sequence diagram was made (Figure 4). The influence degree was high to low: myelosuppression, length of stay, age, diabetes, combined chemotherapy, surgery history, and hormone application. Taking the above seven independent variables as input elements and pulmonary infection as output elements, a three-layer feedforward artificial BP neural network (ANN) model is directly constructed. In the input layer, there were 7 neural nodes; in the hidden layer, there were 7 changeable nodes (hyperbolic tangent transfer function); in the output layer, pulmonary infection occurred during chemotherapy (softmax transfer function). The transfer function of hidden layer was Tansig, the transfer function of output layer was Purelin, the target error is 0.01, the learning rate is 0.1, and LM optimization algorithm is used for network training.

### 3.3. Model Prediction

The area under the ROC curve of ANN was 0.897, which was larger than that of the LR regression model (0.729), indicating that the ANN model has higher predictive ability than the traditional LR model (Figure 5). The results showed that the accuracy, sensitivity, and Youden's index of the ANN model were higher than those of the LR model, but the specificity of the ANN model was lower than that of the LR model (Table 3).

## 4. Discussion

The causes of infection in patients with lung cancer during chemotherapy are complex, and there are various risk factors of infection [18, 19]. Nosocomial infection not only affects treatment and rehabilitation, prolongs hospital stay, and increases medical costs but also significantly affects prognosis and even endangers life. Most of them were elderly patients with age-related organ dysfunction, low immunity, high incidence of multiple diseases, and being easy to complicate with all kinds of hospital infection. The incidence of nosocomial infection was 19.0% (76/40), which was similar to that reported in a domestic literature. Further analysis showed that age≧60 years, length of stay≧14 d, surgery history, combined chemotherapy, myelosuppression, diabetes, and hormone application were risk factors of infection in lung cancer patients during chemotherapy [20].

This study attempts to establish a specific mathematical model by using the risk factors of infection during chemotherapy, evaluating and predicting the possible infection of elderly patients with lung cancer, and evaluating and exploring a new method to predict individual disease. LR is simple and easy to use. It is the most commonly used method to predict the disease status with precise classification. However, it requires that the data meet certain conditions; that is, the dependent variable is a classification variable, the independent variables are independent of each other, and there is no obvious collinearity and interaction, so it is difficult to predict the infection of individual patients effectively. ANN has no requirements for the distribution and type of variables. It is good at dealing with nonlinear, fuzzy, and noisy data. It provides a new way to solve complex medical problems and has been paid more and more attention by medical workers in disease prediction. Relevant research shows that the BP neural network is much better than the traditional Cox regression and LR model for data fitting [21–23].

In this study, the risk factors screened by conditional LR regression analysis were used to establish LR and ANN prediction models, and test samples were used to test. The results show that the accuracy, sensitivity, and Youden's index of the ANN model are better than those of the LR model. In this study, the ROC curve was used to evaluate the predictive effect of the three models. The ROC curve can directly observe the relationship between sensitivity and specificity. The larger the area under the curve, the greater the accuracy of the diagnostic test. The results showed that the area under the ROC curve of the LR prediction model was 0.729 ± 0.084. The area under the ROC curve of the BP neural network was 0.897 ± 0.045, which indicated that the ANN prediction model had better prediction and discrimination performance than the LR prediction model. The data fitting of ANN was better than that of the traditional LR prediction model.

Accurate prediction of lung infection in lung cancer patients undergoing chemotherapy is helpful to improve the treatment effect of patients. Once it is determined that some patients are prone to pulmonary infection, we should pay more attention in clinical work and implement intervention nursing measures. It mainly includes the following: (1) the long-term bedridden patients should help to take the semireclining position during the day, guide effective cough and expectoration, and carry out respiratory function exercise, so as to prevent the occurrence of pneumonia; (2) when eating, the patient should take the sitting position and lie flat after eating for 1 hour to avoid aspiration; (3) encourage patients to exercise in bed and turn over regularly; (4) for patients with nutritional risk, the reasons of loss of appetite or inability to eat should be evaluated in time, and the pretreatment before chemotherapy and the observation and treatment of side effects after chemotherapy should be done well; (5) the ward environment, air circulation, and air conditioning should be deeply cleaned before use, to prevent the spread of bacteria through the air; (6) strict aseptic technical operation should be performed, according to the norms of the implementation of a variety of pipe care; and (7) strengthen oral care and guide patients to gargle after meals, and observe whether there are food residues in the mouth and the changes of oral mucosa.

Because this study is a retrospective study, the definition of patients with infection mainly depends on the doctor's diagnosis, course of disease records, imaging examination, and access to the test sheet in the case with specimen records, including sputum, blood, urine specimens, and pleural effusion. There are still some cases of antibiotic use. Because there are no precise diagnosis and no relevant laboratory and imaging evidence, it cannot determine whether antibiotics in this patient is preventive or therapeutic. This may lead to information limitations and bias, resulting in defects in the established prediction model.

## 5. Conclusions

This study analyzed infection risk factors in patients with lung cancer during palliative chemotherapy. The ROC curve shows that the area under the ROC curve of ANN is more significant than that of LR, which indicates that the prediction ability of ANN is higher than that of the traditional LR model. In the future, more deep learning algorithms [24–26] will be used for predictive analysis of lung cancer.

## Figures and Tables

**Figure 1:** The CT image (a) and pathology (b) from a patient with small-cell lung cancer.

**Figure 2:** Schematic diagram of BP neural network algorithm.

**Figure 3:** BP neural network algorithm flow.

**Figure 4:** Sensitivity analysis of ANN input variables.

**Figure 5:** ROC curve of ANN and LR model for predicting pulmonary infection.

**Table 1:** Demographic characteristics of 400 patients with lung cancer.

Observation items	Features
Age	67.4 ± 15.2
Gender (male/female)	279/121
Cytological type (case)	
Small cell	38
Adenocarcinoma	152
Squamous cell carcinoma	176
Other	34
TNM staging	
IIIA	65
IIIB	131
IIIC	164
IV	40
Nosocomial infection (cases)	
Infected	76
Noninfected	354

**Table 2:** Multivariate analysis of risk factors of infection in patients with lung cancer during chemotherapy.

Factor	*β*	SE	Wald	*P*	OR	95% CI
Age≧60 years	0.718	0.242	9.235	0.004	2.079	0.279-3.182
Length of stay≧14 d	1.349	0.381	14.526	<0.001	3.674	2.138-4.943
Surgery history	0.192	0.064	8.927	0.035	1.207	1.039-1.274
Combined chemotherapy	0.593	0.158	6.142	0.008	1.536	1.123-2.149
Myelosuppression	-1.452	0.017	11.472	<0.001	0.261	0.225-0.493
Diabetes	0.674	0.135	7.243	0.006	1.894	1.492-2.768
Hormone application	0.269	0.114	3.125	0.022	1.347	1.193-1.752

**Table 3:** Evaluation indexes of the ANN model and logistic model.

Model	AUC	Sensitivity	Specificity	Youden's index
LR	0.729 ± 0.084	53.3	92.3	45.6
ANN	0.897 ± 0.045	93.3	86.2	79.5

## Data Availability

The data used to support the findings of this study are available from the corresponding author upon request.
